# Dynamic expression and regulatory mechanism of TGF-β signaling in chicken embryonic stem cells differentiating into spermatogonial stem cells

**DOI:** 10.1042/BSR20170179

**Published:** 2017-07-07

**Authors:** Qisheng Zuo, Kai Jin, Yani Zhang, Jiuzhou Song, Bichun Li

**Affiliations:** 1 Key Laboratory of Animal Breeding Reproduction and Molecular Design for Jiangsu Province, College of Animal Science and Technology, Yangzhou University, Yangzhou, Jiangsu 225009, P.R. China; 2 Animal and Avian Sciences, University of Maryland, Baltimore, MD 20741, U.S.A.

**Keywords:** Embryonic stem cells, Primordial germ cells, RNA-seq, Spermatogonial stem cells, TGF-β signaling

## Abstract

The present study investigated the dynamic expression and regulatory mechanism of transforming growth factor β (TGF-β) signaling involved in embryonic stem cells (ESCs) differentiation into male germ cells. Candidate genes involved in TGF-β signaling pathway were screened from RNA-sequencing (RNA-seq), which were further validated by quantitative real-time PCR (qRT-PCR). Bone morphogenetic protein 4 (BMP4) was used to induce differentiation of ESCs *in vitro*. Inhibition of TGF-β signaling pathway was reflected by Western blot of SMAD2 and SMAD5 expression. Differentiating efficiency of germ cells was evaluated by immunofluorescence and fluorescence-activated cell sorting (FACS). Germ cell marker genes were assessed by qRT-PCR in the differentiation process, with activation or inhibition of TGF-β signaling pathway. In the process of *in vitro* induction, SMAD2 and SMAD5 were found to significantly up-regulated in BMP4 group versus the control and inhibition groups after 4 and 14 days. Expression of *CKIT, CVH, DAZL, STRA8*, and *INTEGRIN α6* were significantly increased in the BMP4 group compared with the control group, while down-regulated in the inhibition groups. The proportion of germ cell-like cells was decreased from 17.9% to 2.2% after 4 days induction, and further decreased from 14.1% to 2.1% after 14 days induction. Correspondingly, expression of marker genes in germ cells was significantly lower. *In vivo* inhibition of TGF-β signaling pathway reduced germ cells formation from 5.5% to 1.6%, and down-regulated the expression of *CKIT, CVH, DAZL, STRA8*, and *INTEGRIN α6*. In conclusion, our study reveals the mechanism regulating spermatogonial stem cells (SSCs) and lays the basis for further understanding of the regulatory network.

## Introduction

Spermatogonial stem cells (SSCs), the basis for spermatogenesis in males, are the only adult stem cells known to pass male genetic information to the next generation [1]. However, the mechanism of differentiation is unclear and germ cell induction efficiency is very low. Therefore, understanding the differentiation of embryonic stem cells (ESCs) into the male reproductive cells is important to offer a theoretical basis for male infertility treatment and regenerative therapy. A variety of intracellular cytokines and the extracellular matrix regulate the process of ESCs differentiation into SSCs, which directly or indirectly contribute to germ line development through different signaling pathways. Previous research on the regulatory signaling pathways has given a preliminary understanding of these mechanisms. For example, some signaling pathways, such as transforming growth factor β (TGF-β)/bone morphogenetic protein (BMP), NOTCH, and WNT, have been reported to regulate physiological behaviors of SSCs (Table 1) [2]. However, to date, no study has systematically profiled the regulatory signaling networks involved in differentiation of ESCs into SSCs.

**Table 1:** Signaling pathways regulating germ cell fate

Molecule	Signaling pathway	Physiological role	Reference(s)
*BMP4*	Smad4/5	Specialized and migration of primordial germ cell (PGC), proliferation, and differentiation of SSCs	Pellegrini et al. (2003)
*GDF9*	Smad4/5	Migration and the elongation of circular sperm	Kawase et al. (2004)
*TGFΒ2*	Smad2/3	The proliferation and differentiation of SSCs	James et al. (2005)
*ACTIVIN*	Smad2/3	SSCs self-renewal	He et al. (2007)
*NODAL*	Smad2/3	PGCs specialized, SSCs self-renewal	He et al. (2007)
*RA/CYP26B1*	RA	The formation and differentiation of SSCs	MacLean et al. (2007)
*WNT3A*	Wnt, Bmp	PGCs specialized	Ohinata et al. (2009)
*NOTCH1*	Notch	The proliferation and differentiation of SSCs	Dirami et al. (2001)
*JAGGED/DELTA*	Notch	The formation and differentiation of SSCs	Dirami et al. (2001)
*UPD (UNPAIRED)*	JAK/STAT	SSCs self-renewal	Tulina and Matunis (2001)
*GDNF*	PI3K/Akt, Ras/Erk1/2, Src	Self-renewal and differentiation of SSC	Trupp et al. (1999)
*SCF*	PI3K/Akt, Ras/Erk1/2, Kit-L	Formation, proliferation, and differentiation of SSC	Feng et al. (2000)
*FGF2*	PI3K/Akt	The proliferation and differentiation of SSCs	Kubota et al. (2004)
*ECM*	Integrin, FAK, MAPK	The formation and proliferation of the SSCs	Dolci et al. (2001); Yoon and Seger (2006)
*DHH/PTC1*	Hedgehog	Spermatogenesis	Clark et al. (2016)

Our previous RNA-sequencing (RNA-seq) data [3] indicated that the *TGF-β* signaling pathway was involved in the development of SSCs from ESCs. The *TGF-β* super family is composed of three subgroups of conserved proteins, including *TGF-βs, BMP*s, and *ACTIVIN* [4]. *SMAD*s are the major downstream signaling molecules [5]. In previous studies, *TGF-β2* was found to variously express in different stages of mouse testis development. *TGFβRII* knockout confirmed the function of TGF-β signaling in regulating the proliferation of germ cells and apoptosis [6]. Meanwhile, *BMP*s have been demonstrated to be essential for germ cell formation [7]. Knockout of *BMP4, BMP8b*, and *BMPZ* resulted in the loss of PGCs [8]. Furthermore, *SMAD4* was found to be widely expressed in the cytoplasm of germ cells, and may regulate testicular development and spermatogenesis through BMP signaling [9]. Although recent advances show the importance of TGF-β signaling in the maintenance of SSCs, the regulation mechanism of the process of ESCs differentiation into SSCs remains unclear. However, exploring the mechanisms of SSCs development thoroughly is logistically difficult. Nevertheless, the differentiation of chicken ESCs into SSCs provides an ideal model to investigate the molecular mechanisms of germ cell cytogenesis, proliferation, and differentiation. In the present study, we explored the dynamic expression and regulatory mechanism of the TGF-β signaling pathway that was identified in our previous study [3] of chicken ESCs differentiation into SSCs. This study lays the foundation for further exploration of the regulatory network involved in germ cell differentiation, and provides the basis for revealing the mechanism of germ cells formation.

## Results

### Isolation, culture, purification, and identification of ESCs, PGCs, and SSCs

In the present study, we used only cultures of the same type of male cells. Sex determination in chickens can be achieved by identification of the chromo-helicase-DNA binding gene on chromosome W (*CHD-W*) that is present only in females (Figure 1A). Fluorescent inverted microscope visualization suggested that ESC clones resemble a bird’s nest with clear edges. PGCs were larger than ESCs with more obvious nuclei and clearly visible areas around the cells. SSCs were large and clumped masses that resembled a bunch of grapes (Figure 1B). Marker gene expression in ESCs, PGCs, and SSCs was identified by quantitative real-time PCR (qRT-PCR). *NANOG, SOX2*, and *OCT4* (totipotency marker genes) were all expressed in ESCs. PGCs expressed *NANOG* and *OCT4*, while SSCs only expressed *OCT4*. Genes that mark germ cells including *CVH, C-KIT, BLIMP1*, and *DAZL* were identified in PGCs and SSCs, while *STRA8*, integrin α6, and integrin β1 were only expressed in SSCs (Figure 1C). All cells were double labeled by antibodies and then sorted using fluorescence-activated cell sorting (FACS) (*n*=3). The proportion of SSEA 1+/Sox2+ cells was 0.88% in ESCs. The proportion of SSEA 1+/C-kit+ cells was 0.71% in PGCs. The proportion of integrin β1+/integrin α6+ cells was 2.43% (Figure 1D).

**Figure 1:** Results are shown for cell isolation, culture, sorting, and identification (**A**) The sex of chicken ESCs and PGCs was determined. Samples 1, 3, 5, 7, 8, and 10 were females of genotype ZW with two DNA fragments at 600 and 450 bp. Samples 2, 4, 6, and 9 were males of genotype ZZ with only one fragment at 600 bp (M: 100 bp marker). (**B**) ESC, PGC, and SSC clones are shown. ESC clones resemble a bird’s nest with clear edges; PGC clones are larger than ESCs with more obvious nuclei and clearly visible areas around the cells; SSC clones are large and clump into a mass that resembles a bunch of grapes, scale bar: 68.8 μm. (**C**) Gene expression in ESCs, PGCs, and SSCs was detected by qRT-PCR. (**D**) Cell sorting results are shown for chicken ESCs, PGCs, and SSCs.

### Differentially expressed genes in the TGF-β signaling network involved in the differentiation of ESCs into SSCs

To analyze the signaling pathways involved in the differentiation of ESCs into SSCs, Venny analysis was performed. A total of 258 signaling pathways were enriched in the process of ESCs differentiation into SSCs (Figure 2A), while 250 signaling pathways were enriched in all the ESCs versus PGCs, PGCs versus SSCs, and ESCs versus SSCs groups (Figure 2B), including the TGF-β signaling pathway. A total of 26 differential expression of genes (DEGs) were enriched in the TGF-β signaling pathway. Three in the ESCs versus PGCs and PGCs versus SSCs groups, and two in the ESCs versus SSCs group were up-regulated. Eleven in the ESCs versus PGCs group, six in the PGCs versus SSCs group, and four in the ESCs versus SSCs group were down-regulated (Figure 2C and D). The values of gene expression and gene ID in the three types of male germ cells were shown in Table 2.

**Figure 2:** Venny analysis of TGF-β signaling pathway genes involved in the process of ESCs differentiation into SSCs (**A**) Cluster analysis of the differential expression of genes (DEGs) in ESCs, PGCs, and SSCs and the DEGs in the key signaling pathway (*P*<0.05). (**B**) Venny analysis of signaling pathways involved in the process of ESCs differentiation into SSCs. (**C**) Twenty-six DEGs in the TGF-β signaling pathway are shown, red represents down-regulated genes, and green represents up-regulated genes. (**D**) Venny analysis for DEG in ESC, PGC, and SSC.

**Table 2:** Gene expression in candidate DEGs in RNA-seq

Name	Gene ID	PGC-RPKM	ES-RPKM	SSC-RPKM
*LOC428957*	XM_426514.2	0.2615316	7.9319858	0.6992365
*TGFBR1*	NM_204246.1	12.03498	35.603308	23.870031
*LOC420783*	XM_418878.2	16.011875	57.815212	27.316224
*ID4*	NM_204282.1	409.18312	23.451504	105.67738
*LOC424261*	XM_422108.2	16.746617	1.1608169	35.198991
*EVC*	NM_001005347.1	6.9683479	1.6706692	14.274811
*THBS1*	XM_421205.2	52.401243	19.336218	258.73535
*TGFBR2*	NM_205428.1	10.809397	0.7589806	9.1517417
*DCN*	NM_001030747.1	77.117439	0.347929	252.23439
*SMAD3*	NM_204475.1	44.019642	6.7470138	59.564046
*TGFB2*	NM_001031045.1	13.271512	2.0175816	12.869093
*SMAD6*	NM_204248.1	74.430471	16.64992	45.766524
*LOC427689*	NM_001039604.1	11.141167	0.5306836	1.2216177
*FST*	NM_205200.1	13.47304	2.0215341	11.959137
*PITX2*	NM_205010.1	32.760948	17.659924	2.5180006
*BMP7*	XM_417496.2	5.1906818	25.747059	1.6204359
*AMH*	NM_205030.1	3.0086921	5.7712117	2769.0292
*NELL2*	NM_001030740.1	16.279439	6.3415645	187.80838
*VWC2*	XM_419028.2	5.0086891	11.553585	68.623922
*SMAD1*	XM_420428.2	32.353393	24.324285	84.278137
*LOC423756*	XM_421631.2	5.1638772	1.6591893	0.3031273
*LOC777130*	XM_001236601.1	659.39145	200.97169	201.94203
*SMAD9*	NM_001024826.1	1.6616052	4.7827217	5.2427059
*LOC417326*	XM_415594.2	0.092275	0.0206579	0.5887629
*LOC421765*	XM_419795.2	0.06848	0.0394222	0.4825528
*E2F5*	NM_001030942.1	9.0192535	11.045055	16.795122

The molecules involved in the TGF-β signaling pathway were classified by their functions, including ligands, receptors, regulators, and downstream molecules. Dynamic expression patterns of the major molecules were shown in Figure 3. In the BMP subgroup, eight ligands were involved in the regulation process. The expression of *BMP4, BMP5, AMH*, and *ADMP* was continuously up-regulated during the differentiation process, while *BMP7* expression was down-regulated. The expression of *GDF6/7, GDF5*, and *VGR1* increased in PGCs, and then decreased slightly when differentiating into SSCs. In the TGF-β subgroup, *TGF-β2* was the only ligand found to vary in expression in different stages of male germ cell differentiation, and its expression increased significantly in PGCs and SSCs compared with that in ESCs. In the *ACTIVIN* subgroup, *INHBA* expression increased from ESCs to SSCs. *NODAL*, a repressor of ESCs differentiation, was down-regulated from ESCs to SSCs. In BMP subgroups, the expression of *BMPRΙA, BMPRΙB*, and *BMPRΙΙ* was largely reduced in PGCs, and increased slightly in SSCs. In the TGF-β subgroup, *TGFβRΙ* expression showed a similar pattern as that in the BMP subgroup, while *TGFβRΙΙ* expression successively increased from ESCs to SSCs. In the Activin subgroup, the expression of *ActivinRI* and *ActivinRII* declined gradually. *SMAD*s are the major regulators in TGF-β signaling. Similar to their receptor *BMPRΙ*, the expression pattern of *SMAD5* and *SMAD9* fluctuated. The expression of SMAD2 and SMAD3 was significantly higher in SSCs than that in ESCs and PGCs, while SMAD6 and SMAD7 expression was increased in PGCs and SSCs. For the downstream molecules, *RBL1* is the negative regulator of cell cycles, and its expression decreased from ESCs to SSCs. Inhibitor of DNA binding (ID) belongs to the dominant-negative helix–loop–helix transcription family. *ID1* and *ID4* were more highly expressed in PGCs than in ESCs. *HISTONE DEACETYLASE, P300*, expression steadily increased throughout the entire differentiation process. The expression of *CMYC*, which is known to drive stem cell self-renewal, gradually declined in PGCs and SSCs. These results strongly indicate that TGF-β signaling is active in the process of ESCs differentiation into SSCs.

**Figure 3:** Dynamic expression patterns of the molecules involved in TGF-β signaling pathway during ESCs differentiation into SSCs Major molecules in the TGF-β signaling pathway were classified based on their functions. The dynamic expression of TGF-β signaling ligands (**A**), receptors (**B**), regulators (**C**), and downstream molecules (**D**) involved in ESCs differentiation into SSCs was derived from the RNA-seq data. Black represents ESCs, Gray represents PGCs, and White represents SSCs.

### Validation of TGF-β signaling pathway-related genes expression in ESCs, PGCs, and SSCs

As shown in Figure 4, 14 genes with major expression differences were selected from the three subgroups for further validation. Results of qRT-PCR confirmed that, from ESCs to PGCs, the expression of *BMP4, TGF-β2, TGFβR2, INHBA, SMAD3*, and *SMAD7* increased, while the expression of *BMPR1A, BMPR1B, TGFβR1, SMAD2, SMAD5*, and *RBL1* decreased. In the differentiation phase of PGCs to SSCs, the expression of *BMPR1A, BMPR1B, TGFβR1, INHBA, SMAD2, SMAD5, SMAD7*, and *RBL1* was up-regulated, whereas the expression of *BMP4, TGF-β2, TGFβR2, ACVR1*, and *MYC* was down-regulated. The qRT-PCR results were consistent with RNA-seq data from our previous study.

**Figure 4:** qRT-PCR validation of key TGF-β signaling genes expressed in ESCs, PGCs, and SSCs Fourteen genes with major expression differences were selected for qRT-PCR validation. (**A**) Ratio of relative expression value of the gene in PGCs versus SSCs. (**B**) The ratio of relative expression values of the genes in PGCs versus SSCs.

### *In vitro* inhibition of TGF-β signaling interfered with SSCs formation

To explore the function of TGF-β signaling in the regulation of male germ cell formation, TGF-β signaling pathway specific inhibitors, LY-100 (100 nM LY2109761—antagonist to the TGF-β subgroup) and LDN-100 (100 nM LDN193189—antagonist to the BMP subgroup), were added to the BMP4 induction medium. Western blot assays showed that expression of SMAD2 and SMAD5 was significantly increased in the BMP4 group on days 4, and was dramatically decreased in the corresponding inhibition groups. Moreover, the expression of SMAD2 and SMAD5 in the double inhibition group was further reduced compared with the single inhibition groups (Figure 5). Concurrently, we found that the expression of *SMAD2* and *SMAD5* was significantly down-regulated.

**Figure 5:** Inhibition efficiency of TGF-β signaling *in vitro* Western blot and qRT-PCR were performed to evaluate the inhibition efficiency of TGF-β signaling *in vitro*. (**A**) Smad2 and Smad5 expression in control and inhibition groups on differentiation days 4 and 14 (CON: control group; LY-100༚100 nM TGF-β subgroup inhibitor LY2109761; LDN-100: 100 nM BMP4 subgroup inhibitor LDN193189). (**B**) Quantitative evaluation of Smad5 expression in different groups on differentiation days 4 and 14. Statistical difference was assessed by comparing the BMP4 group with the control group, and the sample treated with H_2_O was regard as Blank Control (*P<0.05, **P<0.01).

In the BMP4 group, numerous embryoid bodies appeared on day 4, and a few spermatogonial stem-like cells appeared between day 12 and 14. In contrast with the BMP4 induction group, the cells in the LY-100 group and LDN-100 groups displayed no changes on day 4, a few embryoid bodies were observed on day 10, whereas no spermatogonial stem-like cells were seen on or after day 14. Instead, many mast cells were observed in the double suppression group, which were positively stained by Toluidine Blue on day 14 (Figure 5A). Immunofluorescence performed on day 14 showed that a large amount of cells in the BMP4 group expressed *INTEGRIN α6, INTEGRIN* *β1, DAZL*, and *CKIT*, while only a small proportion of CKIT positive cells were observed in the single inhibition group (Figure 6B).

**Figure 6:** Morphology and cell marker identification of the BMP4-induced male germ cells differentiation (**A**) Morphological changes in the cells under BMP4 induction with or without TGF-β signaling inhibitors (LY: TGF-β subgroup inhibitor LY2109761; LDN: BMP4 subgroup inhibitor LDN193189; DOUBLE: two inhibitors were used). Toluidine Blue was used to stain the mast cells in the DOUBLE inhibition group, scale bar: 68.8 μm. (**B**) Immunocytochemical staining of the germ cell markers was used to identify the germ cells. Integrin α6, integrin β1, DAZL, and C-kit were used as the germ cells markers.

Moreover, *CKIT* expression was not detected in the double inhibition group. Expression of the germ cell marker genes, evaluated by qRT-PCR, was significantly increased in the BMP4 group compared with the control group; however, the same germ cell marker genes showed no obvious changes in the inhibition groups (Figure 7A). With FACS, we confirmed that the percentage of CKIT positive cells in the BMP4 group was 17.9% on day 4. However, in the control and inhibition groups, only a small amount of CKIT positive cells (CON: 1.7%; BMP4 + LY-100: 2.5%; BMP4 + LDN-100: 2.8%; and BMP4 + DOUBLE: 2.2%) were counted (Figure 7B and C). On day 14, the percentage of INTEGRIN α6 positive cells in the inhibition groups (BMP4 + LY-100: 3.3%; BMP4 + LDN-100: 2.5%; and BMP4 + DOUBLE: 2.1%) was significantly lower than that in the BMP4 group (14.1%) (Figure 7B and D). The result of haploid generation efficiency detection shown that the percentage of haploid in BMP4 group from 21.7% (BMP group) down to 14.9% (BMP4 + LY-100), 10.5 % (BMP4 + LDN-100), and 8.17% (BMP4 + DOUBLE), when LY-100 and LDN-100 were added into the induced system (Figure 8). These results demonstrated that induction of ESCs to SSCs could be sufficiently blocked by inhibition of the TGF-β signaling pathway *in vitro*.

**Figure 7:** Evaluation of the germ cell marker genes expression *in vitro* by qRT-PCR and FACS (**A**) Expression of germ cell marker genes, including C-Kit, CVH, DAZL, STRA8, integrin α6, and integrin β1 in different treatment groups was evaluated by qRT-PCR. Expression relative to β-actin is presented. (**B**) The PGC marker C-kit and the SSC marker integrin α6 were used to identify the male germ cells with FACS. A positive rate was shown in each group. (**C**) Quantification of the C-kit positive rate in each group based on FACS analysis. (**D**) Quantification of the integrin α6 positive rate in each group based on FACS analysis. Statistical significance was assessed by comparing the BMP4 group with the control group, and the other groups with the BMP4 group (*P<0.05, **P<0.01). The expression of genes in BMP4 group was regarded as positive Control, and the sample treated with H_2_O were regarded as Blank Control.

**Figure 8:** Haploid generation on day 14 during *in vitro* induction The result of haploid generation efficiency detection showed that the percentage of haploid in BMP4 group from 21.7% (BMP group) down to 14.9% (LY-100 group), 10.5 % (LDN-100 group), and 8.17% (DOUBLE group), when LY-100 and LDN-100 were added into the induced system. Quantitative evaluation of haploid efficiency in different groups on differentiation day 14 (capital letters represent high significant differences).

### *In vivo* inhibition of TGF-β signaling impeded ESCs differentiation into SSCs

To further verify the regulatory mechanism of TGF-β signaling in germ cell generation *in vivo*, LY-100 and LDN-100 were injected into *chicken* blastoderms as described previously. Western blot assays confirmed that the expression of SMAD2 and SMAD5 in the LY-100 and LDN-100 groups was significantly suppressed compared with the control group. Meanwhile, the expression of *SMAD2* and *SMAD5* in the double inhibition group was even lower than in the single inhibition group (Figure 9A and B).

**Figure 9:** Inhibition efficiency of TGF-β signaling *in vivo*. qRT-PCR and Western blot were performed to evaluate the inhibition efficiency of TGF-β signaling *in vivo* (**A**) The expression of Smad2 and Smad5 in different groups on embryo development days 5.5 and 18 by Western blot. (**B**) Quantitative evaluation of the expression of Smad2 and Smad5 in different groups on embryo development days 5.5 and 18. Statistical significance was assessed by comparing each group with the control group (*P<0.05, **P<0.01). The expression of Smad2 and Smad5 in Normal incubation process were regarded as Control, and the sample treated with H_2_O was regarded as Blank Control.

The expression of germ cell marker genes was evaluated by qRT-PCR on days 5.5 and 18. The expression of *CKIT, CVH, DAZL, STRA8*, and *INTEGRIN α6* decreased significantly in the inhibition groups versus the control and blank groups. There was no difference between the double and single inhibition groups. Expression of *INTEGRIN β1* did not change across different groups (Figure 10A). FACS analysis showed that, on day 5.5, the amount of CKIT positive cells in the inhibition group was significantly reduced (CON: 12.9%; LY-100: 7.3%; LDN-100: 9.5%; and DOUBLE: 5.4%) (Figure 10B and C), while the number of INTEGRIN α6 positive cells in the inhibition group decreased dramatically on day 18 (CON: 5.5%; LY-100: 3.3%; and LDN-100: 3.6%) (Figure 10B and D). In addition, the proportion of INTEGRIN α6 positive cells in the double inhibition group (DOUBLE: 1.6%) was even smaller than in the single inhibition groups. These results suggested that inhibition of TGF-β signaling arrests the differentiation of ESCs into SSCs.

**Figure 10:** Evaluation of the expression of germ cells marker genes *in vivo* by qRT-PCR and FACS (**A**) Expression of germ cell marker genes, including C-Kit, CVH, DAZL, STRA8, integrin α6, and integrin β1, in different treatment groups was evaluated by qRT-PCR. Their expression relative to β-actin is presented. The expression of genes in Normal incubation process was regarded as Control, and the sample treated with H_2_O was regard as Blank Control (**B**). The PGC marker C-kit and the SSC marker integrin α6 were used to identify the male germ cells with FACS. The positive rate was shown in each group. (**C**) Quantification of the C-kit positive rate in each group based on FACS analysis. (**D**) Quantification of the integrin α6 positive rate in each group based on FACS analysis. Statistical significance was assessed by comparing each group with the control group (*P<0.05, **P<0.01).

## Discussion

TGF-β signaling is known to perform pivotal functions in the differentiation, proliferation, migration, and apoptosis of reproductive cells. In the present study, we analyzed RNA-seq data [3] to profile the dynamic expression pattern of signaling pathways involved in the differentiation of ESCs into SSCs. We identified that TGF-β signaling plays a key role in inducing ESCs differentiation into SSCs. In the BMP subgroup, eight molecules, including *BMP4, BMP5, SMAD5*, and *SMAD9*, were involved and in the TGF-β subgroups, *TGF-β2, TGFβR2, SMAD2*, and *SMAD3* were found to be involved in the regulation of SSCs formation.

BMP4 is a multifunctional cytokine belonging to the TGF-β superfamily. It is released from early the extraembryonic ectoderm, and performs a fundamental function in reproductive cells [10]. Dudley [11] revealed that the production of PGCs was affected by BMP4. Shimasaki [12] observed that the synergistic effect of BMP4 and BMP8b promoted primordial germ cell (PGCs) formation in epiblasts. Toyooka [13] co-cultured the M15 cells that persistently expressed BMP4, with ESCs isolated from *Mvh* transgenic mice and derived sperms differentiated from the ESCs. Subsequently, several studies have attempted to induce ESCs differentiation to male germ cells by BMP4 [14,15]. However, in their study, the male germ cell induction efficiency was low and the characterization of the cells acquired was not sufficient. More importantly, the mechanism by which BMP4 regulates germ cell formation had not been elucidated. In our previous study, different concentrations of BMP4 were used to induce ESCs to differentiate into SSCs, and the optional concentration was determined at 40 ng/ml [16]. Compared with the control group, germ cells appeared after 12 days with a 40 ng/ml BMP4 induction, and the cell number expanded after 2 days. As previously reported, *CVH* is one of the marker genes for SSCs. *DAZL* and *STRA8* are able to initiate the process of meiosis, and *CKIT* is largely expressed in PGCs. *INTEGRIN Α6* is one of the markers for SSCs*.* We identified the cells by immunocytochemical staining of the above-mentioned markers, and confirmed that the cells we acquired possessed germ cell-like characteristics.

*TGF-β1, 2*, and *3* were expressed in mouse fetal testis. Analysis of functional defects in mouse testes revealed that *TGF-β1* mutant mice had a decreased number of germ cells at birth. *TGF-β2* mutant mice had a decreased number of seminiferous cords [17]. Mutations in *BMP7, BMP8A, BMP8B*, or *BMP4* were also observed to block spermatogenesis [18]. In our study, single or double TGF-β signaling inhibitors were injected into chicken embryos. Expression of the germ cell markers in the inhibition group at day 5.5 in the genital ridge and day 18 in the testis was significantly suppressed. FACS analysis revealed that the proportions of PGCs marked by *CKIT* and SSCs marked by *INTEGRIN Α6* were also significantly reduced after *TGF-β* signaling inhibition. Therefore, we further confirmed the role of the TGF-β signaling pathway in germ cell differentiation. In BMP4-induced germ cell formation assays, spermatogonia-like cells appeared 14 days after induction. However, those cells were no longer visible at 14 days after TGF-β inhibition, and the quantity of CKIT positive PGCs and INTEGRIN α6 positive SSCs also decreased dramatically. Hence, the *in vitro* BMP4 induction assay further demonstrated that activation of the TGF-β signaling pathway was necessary to promote SSCs differentiation and production. These results are supported by a study by Chen et al. [19] showing that an Smad-dependent pathway is also involved in retinoic acid-induced germ cell differentiation in mouse ESCs. The results showed treatments of ovaries with BMP4 resulted in a significant (*P*<0.05) increase on the primordial-to-primary follicle transition. The oocytes of primordial follicles treated with BMP4 were also less likely to undergo apoptosis. *TGF-β1, 2*, and* 3* were observed to express in mouse fetal testis. Analysis of functional defects in mouse revealed that TGF-β is required for testicular development [17]. Mutations in *BMP7, BMP8A, BMP8B*, or *BMP4* can block spermatogenesiss [18]. Therefore, we further confirmed the role of TGF-β signaling in germ cell differentiation. BMP4 was used to induce germ cell differentiation *in vitro*, and it is reported that spermatogonia-like cells can be observed after 14 days induction [16]. However, those cells were no longer observed at day 14 after TGF-β inhibition, and the quantity of CKIT positive PGCs and INTEGRIN α6 positive SSCs also decreased dramatically. The *in vitro* BMP4 induction assay further demonstrated that activation of TGF-β is necessary in promoting male germ cell differentiation and production.

Interpretation of the present study is limited by the use of germ cell markers, as cells marked by *DAZL, STRA8, INTEGRIN α6*, and *INTEGRIN β1* were not only confined to be SSCs after 14 days of induction. Therefore, we further detected the efficiency of haploid formation in each of these groups to precisely illustrate the effect of inhibitors on the differentiation of ESCs into SSCs. The results showed that BMP4 can significantly induce ESCs to SSCs differentiation and a small number of cells went into meiosis, indicating the increase in haploid formation efficiency. At this time point, the expression of *DAZL* and *STRA8* was high. When the inhibitors of the TGF-β signaling pathway were added, it showed a decrease in haploid generation efficiency, and the expression of *DAZL* and *STRA8* was low in contrast with the BMP4 induction group. These results were consistent with the normal physiological processes.

In conclusion, the TGF-β signaling pathway is influential in directing the differentiation of ESCs into SSCs. Our study contributes toward revealing the mechanism of regulating SSCs formation, and lays the foundation for further construction of the regulatory networks involved in this process.

## Materials and methods

### Ethics statement

All procedures involving the care and use of animals conformed to U.S. National Institute of Health guidelines (NIH Pub. No. 85-23, revised 1996) and were approved by the Laboratory Animal Management and Experimental Animal Ethics Committee of Yangzhou University.

### Materials

Eggs were collected shortly after fertilization from the poultry institute of the Chinese Academy of Agricultural Sciences Experimental Poultry Farm. A total of 18,340 eggs were collected and used for isolation of three different experimental groups: (1) ESCs, which were used immediately, and (2) PGCs, and (3) SSCs, which were both incubated at 37°C and 75% relative humidity for 5.5 and 18 days respectively, prior to use.

Dulbecco’s modified eagle medium (DMEM) and fetal bovine serum (FBS) were obtained from Gibco (U.S.A.). Mitomycin-C was obtained from Roche. β-Mercaptoethanol, chicken serum, L-glutamine, sodium pyruvate, trypsin, collagen enzyme I, human stem cell factor (HSCF), basic fibroblast growth factor (BFGF), human insulin-like growth factor (HIGF), and murine leukemia inhibitory factor (mUF) were acquired from Sigma–Aldrich. Antibodies specific to the following proteins were purchased: SSEA-1 (Biolegend, San Diego, CA, U.S.A.; dilution ratio 1:1000), Sox2 (abcam, Cambridge, England; dilution ratio 1:1000), SSEA1 (abcam, Cambridge, England; dilution ratio 1:1000), C-kit (SouthernBiotech, Birmingham, AL, U.S.A.; dilution ratio 1:1000), integrin α6 and integrin β1 (Millipore; dilution ratio 1:1000), and goat anti-mouse IgM (flourescein isothyocyanate [FITC] labeled; Bio-Synthesis, Inc., Texas, U.S.A.; dilution ratio 1:1000).

### Methods

#### Isolation and culture of ESC, PGC, and SSC

Separation and cultivation of ESCs, PGCs, and SSCs were performed as described previously [14–16].

#### Sex determination

Genomic DNA from ESCs and PGCs was extracted to identify the sex of the germ cells through polymerase chain reaction (PCR) amplification using the primer sequences: F: GTTACTGATTCGTCTACGAGA and R: ATTGAAATGATCCAGTGCTTG. The PCR cycle consisted of 30 cycles of 98°C for 10 s, 49°C for 5 s, 72°C for 30 s followed by long-term storage at 4°C. Only male germ cells were used in RNA-seq analyses.

#### Flow cytometry cell sorting

Highly purified cells were acquired through cell sorting using two antibodies in combination to label and select cells. Antibodies to SSEA-1(dilution ratio 1:1000) and Sox2 (dilution ratio 1:1000) were used to identify ESCs, antibodies to C-kit (dilution ratio 1:1000) and SSEA-1 (dilution ratio 1:1000) were used to identify PGCs, and antibodies to the α-6 and β-1 integrins (dilution ratio 1:1000) were used to identify SSCs.

#### RNA-seq and analysis

ESCs, PGCs, and SSCs were collected by cell sorting, total RNA of which were extracted according to mirVana™ RNA Isolation Kit (Applied Biosystem p/n AM1556) kit, and total RNA was purified using QIAGEN RNeasy™ Kit. Illumina Inc.’s (U.S.A.). mRNA-seq procedures were followed for RNA-seq. A total of 50 ng of cell tissue was sequenced using the HiSeq 2000 system (Illumina, Inc., U.S.A.) by Shanghai OE Biotech. Co., Ltd. Results were compared against the database to obtain annotations for every identified gene. An enrichment analysis of the significance of gene ontology (GO) function and pathway was based upon the log2 value of the DEGs by DAVID (http://david.abcc.ncifcrf.gov/home.jsp), FunNet (http://www.funnet.info/), and WEGO (http://wego.genomics.org.cn/cgi-bin/wego/index.pl). Hierarchical cluster was conducted by the Eisende Cluster based upon the log2 value of the DEGs. The distance of the hierarchical clusters was determined by Euclidean distance and calculated by mean distance. The regulating network of candidate key genes was analyzed by the FUNNET database (http://www.funnet.info/). The data of RNA-seq were uploaded to the SPA database, and the reference numbers are SRR3720923, SRR3720924, and SRR3720925.

#### *In vitro* mutagenesis

The 2-d development stage of the ESCs was selected for the experiment following the methods established in previous work [20]. Cells were seeded into 24-well plates with a cell density of 10^5^ cells per well. Cell treatment groups were as follows: control group: with no treatment; BMP4 group: induction with 40 ng/ml BMP4; LY-100 group: induction with BMP4 and 100 nM LY2109761; LDN-100 group: induction with BMP4 and 100 nM LDN193189; DOUBLE group: induced with BMP4 and equal concentrations of both of the inhibitors. The gene expression of *C-KIT, DAZL*, integrin α6, and integrin β1. Smad2, Smad5, and Notch1 were detected by qRT-PCR and Western blot. LDN-193189 (Gene Operation, ITB1003-0002MG, U.S.A.) is inhibitor for TGF-β/Smad; LY2109761(Gene Operation, ITB1006-0002MG, USA) is inhibitor for TGF-β/Smad.

#### Chicken embryo injections

Fertilized embryos were grouped as follows: blank group: without any treatment during the incubation process; control group (CON): injection with 100 μl of ddH_2_O; LY-100 group: injection with 100 μl of LY2109761 (100 nM); LDN-100 group: injection with 100 μl of LDN193189 (100 nM/l); dual inhibitor group (DOUBLE): injection with 50 μl of LDN193189 (200 nM); and 50 μl of LY2109761 (200 nM). Eggs were injected at the top with a TGF-β signaling pathway inhibitor as described previously [21]. They were then sealed with paraffin and incubated at 38.5°C. Samples were collected after 5.5 and 18 days of incubation. Smad2, Smad5, C-kit, Dazl, CVH, and Stra8 gene and protein expression was detected by qRT-PCR and Western blot.

#### qRT-PCR validation

Total RNA was extracted with an RNEasy kit (QIAGEN). Reverse transcription was performed to establish cDNA. qRT-PCR was performed according to the instructions provided in the fluorescence quantitative PCR kit, using SYBR as the fluorescence reagent and a fluorescence ration PCR instrument (7500 System fluorescence quantitative instrument, Applied Biosystems, Carlsbad, California). Data were analyzed using the 2^−ΔΔ^ *C*_t_ relative quantitative method in Microsoft Excel. The primers used are listed in Table 3,4

**Table 3:** Primers information for qRT-PCR in TGF-β pathway

Gene name	Genbank accession number	Primers for qPCR	*T*_m_ (°C)	Size (bp)
*BMP4*	NM_205237	F: TGGTAACCGAATGCTGATGG	58	232
		R: GATGACGGCTGATTTGCTG		
*BMPR1A*	NM_205357	F: GGATTTACAGCCGACAT	58	275
		R: GTAGCCCTGAGCCACT		
*BMPR1B*	NM_205132	F: ATTAGAGGGCTCGGACTT	58	246
		R: GCTTCTTGCCGCTTG		
*BMPRII*	NM_001001465.1	F: AAGGACCCGTATCAGC	59	299
		R: TCAGGAGGTGGGAAGT		
*TGF-β2*	NM_001031045.1	F: AAATGCCATCCCACCA	55	158
		R: GCTCTATCCGCTGCTCC		
*TGFβR1*	NM_204246	F: TGCGGACAACAAAGAC	55	281
		R: GCCTAACTGCCAACCC		
*TGFβR2*	NM_205428	F: GCCTACCGCACTCACA	55	177
		R: TTCAATGGGCAGCAAT		
*INHBA*	NM_205396	F: AGCCGAAAGGCAACTC	55	190
		R: CAGGCAATCCGCACA		
*ACVR1*	NM_204560	F: GGGGTCTTTGTATGACTATCT	60	238
		R: CTGGTTCGTGCTTTGG		
*SMAD2*	NM_204561	F: GCCATTACCACTCAGAAC	55	174
		R: TTTACGATGCGACACCT		
*SMAD3*	NM_204475	F: GGCACATCGGAAGAGGA	55	210
		R: GGTTTACAGACTGAGCCAAGA		
*SMAD5*	NM_001014968	F: TCGCCAAACAGTCCC	55	230
		R: GCAACAGGCTGAACATC		
*SMAD7*	XM_427238.2	F: CAGTTCCTGATGGGTTATGG	55	240
		R: GCTTCTGTTGTCCGAGTTGA		
*RBL1*	XM_417312.2	F: AGATGAAAGCCTCAGAAGA	58	237
		R: CAAAGTCACCCACTGTTAGA		
*MYC*	NM_001030952	F: CCCAGCAAGAACTACGATTACG	55	223
		R: CGGTGGAAGGGAAGCAG		

**Table 4:** Primers information for qRT-PCR detected ESCs differentiation *in vitro*

Gene	Genbank accession number	Primers for qPCR	T_m_ (°C)	Size (bp)
*CVH*	NM_001146142.1	F: TGGTTTCAGAACCAACGAATGAAG	64	180
		R: TGCACTGGTCACAGCCTGAAG		
*CKIT*	D13225.1	F: GCGAACTTCACCTTACCCGATTA	64	150
		R: TGTCATTGCCGAGCATATCCA		
*DAZL*	NM_204218.1	F: TGTCTTGAAGGCCTCGTTTG	61	138
		R: CATATCCTTGGCAGGTTGTTGA		
*INTEGRIN α6*	NM_205289.1	F: GCTGGAAACATGGACCTGGATAA	64	145
		R: TTCAGGTCAAGTTTGTCAGGCTGTA		
*STRA8*	JX204292.1	F: CCACGGCTATTTCACACCTCTG	64	114
		R: GCTCTTGGCAAGCATCCGTA		
*β-ACTIN*	L08165.1	F: CAGCCATCTTTCTTGGGTAT	60	164
		R: CTGTGATCTCCTTCTGCATCC		

#### Western blotting

We collected genital ridges and testes from the chicken embryos unhatched at 5.5 and 18 days, as well as cell groups that were inducted at 4 and 14 days. Then RIPA buffer was used to lyse cells and extract proteins. Protein concentration was determined; 20 μg of total cellular protein was mixed with 5 μl of sample buffer and boiled for 3–5 min to denature the proteins. Proteins were separated by SDS/PAGE (10% gel), and transferred to nitrocellulose membranes, which were then semi-dried and blocked with tris-buffered saline with Tween containing 5% fetal calf serum for 1 h at room temperature. The membranes were incubated in the primary antibodies (SMAD2, SMAD5, and β-ACTIN) overnight at 4°C. After washing by PBS Tween (PBST), the corresponding secondary antibodies were added and incubated at 37°C for 2 h. Bands were visualized using a DAB Substrate Kit to detect horseradish peroxidase.

#### Immunocytochemistry

After induction, cells in 24-well plate were fixed with 4% paraformaldehyde for 30 min, rinsed with phosphate-buffered saline (PBS) three times, and then permeabilized in 0.5% TritonX-100 for 10 min. Cells were then washed with PBS three times and blocked with 10% bovine serum albumen (BSA) in PBS for 30 min at room temperature. The primary antibodies of CKIT (dilution ratio 1:1000), DAZL (dilution ratio 1:1000), INTEGRIN α6 (dilution ratio 1:1000), and INTEGRIN β1 (dilution ratio 1:1000) were added into the cells, and the plate with cells was incubated overnight at 4°C. Samples in 24-well plate were rinsed three times in PBS Tween (PBST) before the corresponding secondary antibody was applied and sections were incubated in the dark at 37°C for 1 h. Samples in 24-well plate were then rinsed three times with PBST, and DAPI was applied to stain the nuclei. Samples were observed using fluorescence microscopy.

#### Haploid generation

The samples of different groups were collected on the 14th day in the induction process, and the cell suspension was made. The cells were sorted by flow cytometry with staining by PI. The experiment was carried out three times, and the difference of haploid efficiency between different groups was analyzed by Spss17.0.

### Statistical analysis

All data are presented as mean ± standard error (*X* ± SEM), and the differences between groups were analyzed by *t*-test and one-way ANOVA. *P* values of 0.05 or less were considered as statistically significant.

## Abbreviations

BFGF: basic fibroblast growth factor
BMP4: bone morphogenetic protein 4
DEG: differentially expressed gene
ESC: embryonic stem cell
FACS: fluorescence-activated cell sorting
GO: gene ontology
HIGF: human insulin-like growth factor
HSCF: human stem cell factor
mUF: murine leukemia inhibitory factor
PBST: PBS Tween
PGC: primordial germ cell
qRT-PCR: quantitative real-time-polymerase chain reaction
RNA-seq: RNA-sequencing
SSC: spermatogonial stem cell
TGF-β: transforming growth factor β
